The article "To be or not to be empathic: the combined role of empathic concern and perspective taking in understanding burnout in general practice" was published in 2014. Journal: BMC Fam Pract.

# To be or not to be empathic: the combined role of empathic concern and perspective taking in understanding burnout in general practice

**DOI:** 10.1186/1471-2296-15-15

**Published:** 2014-01-23

**Authors:** Martin Lamothe, Emilie Boujut, Franck Zenasni, Serge Sultan

**Affiliations:** 1 Department of Psychology, University of Montreal, Succursale Centre- ville, PO Box 6128, Montreal, QC H3C 3J7, Canada; 2 Institute of Psychology, Paris Descartes University, Paris, France; 3 Department of Pediatrics, University of Montreal, Montreal, QC, Canada; 4 Sainte-Justine UHC, Montreal, QC, Canada

**Keywords:** Empathy, Sympathy, Empathic concern, Perspective taking, Burnout, Physicians, General practice

## Abstract

**Background:**

General practice is stressful and burnout is common among family physicians. A growing body of evidence suggests that the way physicians relate to their patients could be linked to burnout. The goal of this study was to examine how patterns of empathy explained physicians’ burnout.

**Methods:**

We surveyed 294 French general practitioners (response rate 39%), measured burnout, empathic concern (EC) and perspective taking (PT) using self-reported questionnaires, and modeled burnout levels and frequencies with EC, PT and their interaction in linear and logistic regression analyses.

**Results:**

Multivariate linear models for burnout prediction were associated with lower PT (β *= −*0.21, p < 0.001) and lower EC (β *= −*0.17, p < 0.05). Interestingly, the interaction (EC x PT) also predicted burnout levels (β = 0.11, p < 0.05). The investigation of interactions revealed that high scores on PT predicted lower levels of burnout independent from EC (odd ratios (OR) 0.37; 95% confidence interval (95% CI) 0.21–0.65 p < 0.001), and high scores on both EC and PT were protective against burnout: OR 0.31; 95% CI 0.15–0.63, p < 0.001).

**Conclusions:**

Deficits in PT alone might be a risk factor for burnout, whereas higher PT and EC might be protective. Educators should take into account how the various components of empathy are potentially associated with emotional outcomes in physicians.

## Background

Burnout is prevalent among physicians worldwide, with estimates of physician burnout ranging from 30 to 70% [1-4]. Physician burnout has serious repercussions, such as deterioration in patient care, medical errors, substance abuse, interpersonal difficulties, depression and suicide [3,5,6]. In a recent survey, 18% of medical residents rated their mental health as either fair or poor, which is more than double that reported in the general population of the same age [7]. Suicide is one of the major causes of early death in physicians, the suicide rate being 1.4 times higher for male physicians and 2.3 times higher for female physicians compared to the average population [8].

The article "To be or not to be empathic: the combined role of empathic concern and perspective taking in understanding burnout in general practice" was published in 2014. Journal: BMC Fam Pract.

The heavy workload of physicians and lack of resources are important risk factors for burnout [9]. Physicians are often overloaded with the demands of caring for patients within constraints of diminished organizational resources. Physicians are also confronted with various emotionally distressing situations associated with illness, dying, fear and suffering, which in turn could result in extremely challenging interactions with patients and other medical staff [5].

Good doctor-patient relationships are fundamental for better health outcomes [10,11]. A meaningful interpersonal relationship with the patient depends on understanding both the patient’s cognitive and affective states [12]. In this context, both empathy and sympathy appear to be crucial components in the doctor-patient relationship [13]. Empathy has been defined as “a cognitive (as opposed to affective) attribute that involves an understanding of the inner experiences and perspectives of the patient, combined with a capability to communicate this understanding to the patient” [14]. Sympathy has been defined as a “predominantly emotional attribute that involves feeling patients’ pain and suffering” [15]. The goal of empathy is to *know* the patient better, while the goal of sympathy is to *feel* the patient’s emotions better [15]. It is important to distinguish the two concepts because they may lead to different outcomes. For example, in hypothetical situations, sympathetic physicians, compared with empathetic ones, have utilized more health care resources in the care of their patients [16]. Some authors believe that empathy leads to personal growth, career satisfaction and optimal clinical outcomes, while sympathy could be detrimental to objectivity in decision making, and lead to compassion fatigue and burnout [13].

A core component of empathy in the context of patient care is perspective taking. It is a cognitive attribute that consists of the effort to adopt the point of view of another person and see things from their perspective [17]. Perspective taking has been shown to increase patient satisfaction [18], as well as physician’s well-being [4]. Empathic concern, which is conceptually closer to sympathy or affective empathy, has been described as an emotional reaction (e.g., compassion) to another individual’s emotional response (e.g., sadness) [19]. It is the emotional reaction of an individual who is attentive to others’ situations and spontaneously engages in prosocial helping behaviors [19,20].

Both perspective taking (i.e., cognitive empathy) and empathic concern (i.e., affective empathy) appear to be playing an important role in physicians’ understanding of their patients. However, while perspective taking has been viewed to be always beneficial in patient care, a too elevated level of empathic concern (or sympathetic feelings) could interfere with objectivity in diagnosis and treatment [21]. Therefore, some *affective distance* between physicians and their patients has been considered desirable to maintain both clinical neutrality and physician’s emotional balance [14].

The article "To be or not to be empathic: the combined role of empathic concern and perspective taking in understanding burnout in general practice" was published in 2014. Journal: BMC Fam Pract.

Data from cognitive neuroscience suggest that empathy incorporates both emotion sharing (automatic, bottom-up information processing) and executive control to regulate the emotional experience (top-down information processing) [22]. Studies have demonstrated that observing another person experience pain activates a large part of the pain matrix in the observer and this in turn could result in empathic concern and sympathy in the observer [22]. However, the same signals could represent a threat for the observer that could ultimately lead to personal distress or compassion fatigue [23]. Thus, regulatory mechanisms must operate in people who are in contact with individuals who are in states of suffering in order to prevent their distress from impairing their ability to help [24]. If physicians fail to regulate their emotions adequately in their interactions with their patients, they may experience feelings of being emotionally drained over time. Physicians’ inability to properly manage their emotions could lead to emotional exhaustion, which is the most obvious manifestation of burnout [9].

The goals of this study were: 1) to identify the contribution of empathic concern (affective empathy) and perspective taking (cognitive empathy) to burnout, beyond the contributions of demographic variables associated with burnout, and (2) to understand how empathic concern, perspective taking and their interaction could predict burnout. We hypothesized that scores indicative of higher physician burnout would be associated with lower perspective taking (cognitive empathy) and higher empathic concern (sympathy) scores, taken individually. Based on previous assumptions, we also expected that higher levels of burnout (or higher risks of extreme burnout) would be associated with high levels of empathic concern combined with lower levels of perspective taking.

## Methods

### Participants

French general practitioners were approached in two ways. The majority (80%) were recruited through the e-mail registry of the French national professional society ‘Société de Formation Thérapeutique du Généraliste’ (professional society for the continuing education of general practitioners). All members of this society were prompted by e-mail to invite physicians to participate in an Internet based survey (with a maximum of two prompts). Physicians were also approached during the yearly national congress for general practice (20%). The inclusion criterion was that the participant needed to be a working general practitioner. There were no criteria regarding age, gender or seniority. Each participant gave written informed consent before the beginning of the study. The study received ethical approval from the institutional ethics committee at the University Paris Descartes. A full description of participant recruitment procedures is available in a previous report [25].

The article "To be or not to be empathic: the combined role of empathic concern and perspective taking in understanding burnout in general practice" was published in 2014. Journal: BMC Fam Pract.

### Measurement of burnout

The widely used Maslach Burnout Inventory (MBI) consists of 22 items that are scored on 7-point Likert scales (0 = never, 6 = everyday). The MBI comprises 3 subscales: emotional exhaustion (score range 0 to 54), depersonalization (score range 0 to 30) and personal accomplishment (score range 0 to 49). High scores on the emotional exhaustion and depersonalization subscales paired with low scores on the personal accomplishment subscale were indicative of high levels of burnout. An example of a positively worded item is, “I feel emotionally drained from my work”. The MBI has been previously validated in samples of health care professionals, including general practitioners, and has been shown to have strong content, internal structure and criterion validity [26-28]. As previously suggested [29], we recoded the personal accomplishment items and summed the 22 items of the MBI to form a single global measure of burnout. This procedure resulted in a highly consistent scale in the present sample (α = .84). We defined extreme burnout as a mean score above the 75^th^ percentile (corresponding to a score of 29) (n = 71).

### Measurement of perspective taking

The Jefferson Scale of Physician Empathy (JSPE) is a 20-item physician self-assessment tool, which evaluates empathy on a 7-point Likert scale (1 = strongly disagree, 7 = strongly agree). Previous studies have suggested that the scale consists of three components: perspective taking, compassionate care and standing in the patient’s shoes [30,31]. A study with the French version of the scale confirmed the three-factor structure of the scale, but did not support the calculation of a global score [32]. We used the perspective taking subscale to evaluate the cognitive aspect of physicians’ clinical empathy. A sample item is, “I try to think like my patient in order to render better care”. Previous studies have evidenced the validity (construct, divergent, convergent, criterion related) and reliability (Cronbach’s alpha, test-retest) of the JSPE among medical students and physicians [12,13,30,32].

The article "To be or not to be empathic: the combined role of empathic concern and perspective taking in understanding burnout in general practice" was published in 2014. Journal: BMC Fam Pract.

### Measurement of empathic concern

The Toronto Empathy Questionnaire (TEQ) consists of 16 items, each rated on a 5-point Likert scale (0 = never, 4 = always), which assesses a single factor of general empathic concern [19]. The TEQ conceptualizes empathy as a primarily emotional process. The scale provides a score ranging from 0 to 64, whereby the higher the score, the higher the self-reported emotional concern. An example of a positively worded item is, “I find that I am ‘in tune’ with other people’s moods”. The TEQ has demonstrated good internal consistency, high test-retest reliability and strong convergent validity [19].

### Statistical analyses

Pearson correlation coefficients were calculated to explore the links between burnout scores, socio-demographic characteristics, perspective taking and empathic concern. A multiple linear regression explored the effects of empathic concern, perspective taking and their interaction on burnout. Further, we performed logistic regressions to compute the odds ratios regarding the presence of extreme burnout associated with perspective taking, empathic concern as well as their interaction. Odds ratios were adjusted for marital status, as this was related to burnout in preliminary analyses. We set the probability of type 1 error at an alpha of .05. SPSS version 19 was used to perform the statistical analyses.

## Results

Of the 81 general practitioners approached during the annual French National Congress of General Practice, 75% completed the questionnaires (n = 61) and of the 680 members of the ‘Société de Formation Thérapeutique du Généraliste’, 36% completed the questionnaires (n = 247). In total, 308 questionnaires were completed. The total response rate was 39%. We excluded 14 questionnaires due to incomplete data. Therefore, the final sample was composed of 294 participants. No statistically significant differences were found between the two sub-samples on any of the variables, and thus the two sub-samples were merged.

The characteristics of the sample are described in Table 1. The description of burnout and empathy scores is reported in Table 2. In preliminary analyses we observed that women had higher levels of emotional exhaustion (N 143, M 18.4, Standard Deviation (SD) 9.6) than men (N 151, M 15.4, SD 10.3) (p < .01 d = .30). They had lower levels of depersonalization (M 6.0, SD 4.8 in comparison to M 7.1, SD 5.1) but higher levels of empathic concern (M = 48.8, SD 5.3 in comparison to M 44.9, SD 5.3) than men (respectively p < .05 d = .23 and p < .001 d = .40). The other dimensions did not differ according to gender. When examining bivariate correlation with burnout, burnout was found to be significantly associated with marital status (living alone) (r = 0.14, p < 0.05), but was not related to other demographics or practice variables. Therefore, following the recommendations of Cohen (1988) we controlled for marital status in subsequent analyses [33]. Burnout was also related with lower scores in perspective taking (r = −0.24, p < 0.01) and empathic concern (r = −0.17, p < 0.01). When looking into components of burnout, higher emotional exhaustion was associated with being a woman (r = 0.15, p < 0.05), living alone (r = 0.12, p < 0.05), and lower JSPE Standing in the Patient’s Shoes (r = −0.14, p < 0.05). There were no significant associations between emotional exhaustion and other empathy measures. Depersonalization was negatively associated with being a woman (r = −0.12, p < 0.05) and all empathy measures (r = −0.18 to −0.32, p < 0.01). Higher personal accomplishment was associated with higher empathy on all empathy measures (r = 0.18 to 0.40, p < 0.01). When predicting burnout in a linear regression model using empathic concern, perspective taking and their interaction as predictors, we observed that each of the predictors was uniquely associated with the outcome, with lower empathy scores predicting higher burnout (model adjusted for marital status). Higher empathic concern (ß = −0.17, p < 0.05) and higher perspective taking (ß = −0.21, p < 0.001) predicted lower burnout. Interestingly, the interaction term was also significant (ß = 0.11, p < 0.05) suggesting a moderating role of empathic concern in the perspective taking – burnout relationship. The total model explained 10% of the variance of burnout (R^2^ = 0.08 without controls). In order to interpret this interaction we plotted burnout levels as a function of empathy patterns determined by median splits and observed that burnout was even lower in participants with high perspective taking scores when empathic concern scores were also lower. To investigate this interaction in a clinically meaningful manner, we explored factors associated with the odds of extreme burnout using a logistic regression model (odds adjusted for marital status, Figure 1). This interaction is well illustrated when comparing the proportion of burnout according to levels in PT and EC (Figure 2). Proportions of participants showing burnout differed according to the combined effects of PT and EC (χ^2^ = 22.74, p < 0.001, Cramer’s V = 0.28). Higher PT could be even more beneficial when participants showed higher EC and higher EC could be beneficial only when participants showed higher PT.

The article "To be or not to be empathic: the combined role of empathic concern and perspective taking in understanding burnout in general practice" was published in 2014. Journal: BMC Fam Pract.

**Table 1:** Characteristics of the sample (N = 294 General practitioners)

	**Men**		**Women**		**Total sample**						
**Variable**	**M/n (%)**	**SD**	**M/n (%)**	**SD**	**M/n (%)**	**SD**	**Mdn**	**Range**	**t/X**^**2**^	**p**	**d/V **^**b**^
**Gender**	151 (51)		143 (49)		294				2.18	< 0.001	
**Age**	53.51	8.69	48.35	9.40	51.00	9.39	52	27–75	4.90	< 0.001	0.57
**Living alone**	14 (9)		42 (29)		56 (19)				19.24	< 0.001	0.26
**Years of clinical experience**	25.58	9.19	19.85	9.77	22.80	9.87	25	1–50	5.19	< 0.001	0.61
**Number of consultation/week**	97.91	32.26	85.63	30.74	91.93	32.07	90	20–200	3.34	< 0.001	0.39
**Length of consultation**											
**< 16 min**	50 (33)		32 (22)		82 (28)				5.12	0.077	0.13
**16-20 min**	76 (50)		77 (54)		153 (52)				5.12	0.077	0.13
**> 20 min**	25 (17)		34 (24)		59 (20)				5.12	0.077	0.13
**Burnout levels**^**a**^											
**Low**	49 (33)		39 (27)		88 (30)				0.94	0.63	0.06
**Average**	97 (64)		99 (69)		196 (67)				0.94	0.63	0.06
**High**	5 (3)		5 (4)		10 (3)				0.94	0.63	0.06

^a^Levels according to the MBI manual guidelines. ^b^Effect sizes for the comparison across genders, Cohen’s d or Cramer’s V.

**Table 2:** Description of psychosocial measures

	**Total Sample**			
**Variable**	**M**	**SD**	**Mdn**	**Range**
**Burnout (MBI)**				
**Emotional exhaustion**	16.86	10.07	15	1–46
**Depersonalization**	6.55	4.98	5	0–24
**Personal accomplishment**	40.15	6.05	41	20–48
**Burnout**	31.26	15.79	29	3–85
**Clinical empathy (JSPE)**				
**Perspective taking**	53.25	7.87	53	20–70
**Compassionate care**	47.72	4.92	47	31–56
**Standing in patients’ shoes**	10.83	2.45	11	2–14
**Total score**	111.81	10.60	112	84–134
**Empathic concern (TEQ)**	45.89	5.37	46	24–58

MBI: Maslach Burnout Inventory; JSPE: Jefferson Scale of Physician Empathy; TEQ: Toronto Empathy Questionnaire.

**Figure 1:** **Perspective Taking, Empathic Concern and their Interaction as Predicting Burnout in 294 French General Practitioners (Odds Ratio Adjusted for Marital Status).** We dichotomized Perspective Taking and Empathic Concern by the median; low Perspective Taking = score ≤ 53, high Perspective Taking = score > 53; low Empathic Concern = score ≤ 46 (n = 151), high Empathic Concern = score > 46 (n = 143). The odds for burnout were significantly lower in participants with high PT (OR 0.37, 95% CI 0.21–0.65, p < 0.001), high EC (OR 0.57, 95% CI 0.33–0.98), p < 0.05) and high on both PT and EC (OR 0.31, 95% CI 0.15–0.63, p < 0.001).

**Figure 2:** **Interaction Between Perspective Taking and Empathic Concern to Explain Burnout Frequencies.** PT = Perspective Taking; EC = Empathic Concern. Perspective Taking and Empathic Concern were dichotomized at the median. Low Perspective Taking = score ≤ 53, n = 153; High Perspective Taking = score > 53, n = 141; Low Empathic Concern = score ≤ 46, n = 151; High Empathic Concern = score < 46, n = 143. We divided the participants into four groups based on the distribution of their empathy scores: (1) low Empathic Concern–low Perspective Taking (n = 99), (2) low Empathic Concern–high Perspective Taking (n = 52), (3) high Empathic Concern–low Perspective Taking (n = 54) and (4) high Empathic Concern–high Perspective Taking (n = 89). Percentage of extreme burnout for low Empathic Concern–low Perspective Taking, low Empathic Concern–high Perspective Taking, high Empathic Concern–low Perspective Taking and high Empathic Concern–high Perspective Taking was 33%, 22%, 32% and 11% respectively.

The article "To be or not to be empathic: the combined role of empathic concern and perspective taking in understanding burnout in general practice" was published in 2014. Journal: BMC Fam Pract.

## Discussion

To our knowledge, this is the first study investigating patterns of empathy in relation to burnout in general practitioners. In line with our hypothesis, we found that a higher level of perspective taking was significantly associated with a lower proportion of burnout in this sample of general practitioners (Figure 1). Contrary to our expectations, we found that a higher level of empathic concern was also significantly associated with a lower proportion of burnout (Figure 2). The odds of experiencing burnout were significantly lower when physicians scored high on perspective taking, high on empathic concern and high on both perspective taking and empathic concern (Figure 1). In our sample, the group of physicians with high levels of both empathic concern and perspective taking had a significantly lower risk of indicating burnout (Figure 1).

The fact that scores indicative of lower burnout were associated with higher perspective taking and empathic concern scores taken individually is in line with previous studies that used the JSPE [34] and the Interpersonal Reactivity Index (IRI) [35] as measures of empathy. An original finding in our study concerned the interaction between perspective taking and empathic concern. We found that empathic concern had no effect when perspective taking was low. However, when perspective taking was high, the burnout percentage was much lower when empathic concern was also high (as summarized in Figure 2). One plausible explanation for this interaction is that empathic concern would be more beneficial to physicians when perspective taking is also high. In other words, it is when physicians are good at adopting the point of view of their patients that their emotional reaction and pro-social helping behaviors reduce the effect of exposure to stress.

In the context of patient care, cognitive empathy (an ability that includes perspective taking) requires effort aimed at understanding the patient’s experiences while keeping a certain affective distance. However, sympathy (or emotional concern) involves a non-conscious and difficult to regulate feeling of sharing in the patient’s suffering [13]. Empathy and sympathy imply different mental activities during information processing. The affective reaction (in sympathy) is influenced by the process of arousal, whereas the cognitive response (in empathy) is influenced by the process of appraisal [36]. It is important to make a distinction between empathy and sympathy, because it has important implications for the physician-patient relationship.

The article "To be or not to be empathic: the combined role of empathic concern and perspective taking in understanding burnout in general practice" was published in 2014. Journal: BMC Fam Pract.

Our results are coherent with a body of research showing that empathy is associated with positive clinical outcomes on various levels: lower emotional distress, higher adherence, lower use of clinical resources, etc. [37-39]. In physicians, cognitive empathy and emotion regulation skills have been recognized as protective factors against stress. Remaining open to the patients’ experience will also lead to better mental health in physicians [18,38]. A recent qualitative study highlighted the importance of physician’s gratification derived from the physician-patient relationship [10]. Physicians reported that showing interest in the patient was one decisive factor protecting them from monotony. Good relationships with patients were reflected in the patients’ gratitude, which in turn was a source of strength for the physician [10]. Our results go a step further suggesting that cognitive empathy but not affective empathy, when used independently, will lead to lower burnout or higher well-being.

Although higher affective empathy did not appear as a risk factor for burnout in this study, we found associations with burnout contrasting with the other kind of empathy. It has been suggested that beyond a certain point affective empathy could actually hinder physician’s performance and affect medical decision-making [30]. Sharing the patient’s emotions (sympathy) can lead to empathic overarousal or personal distress (an aversive self-focused emotional reaction to the apprehension of another person’s emotional state) [22]. Physicians sharing patient’s emotions may have difficulty maintaining a sense of ownership regarding whose emotions belong to whom. To complement the effect of affective empathy, professionals need a high level of emotional regulation skills, as is reflected by high cognitive empathy. Affective sharing without emotion regulation skills may be associated with personal distress, compassion fatigue and burnout [23], which in turn would decrease empathic concern and pro-social helping behavior [21]. This phenomenon could explain the interactive effect of affective empathy (empathic concern) with cognitive empathy (perspective taking) in the present study.

The article "To be or not to be empathic: the combined role of empathic concern and perspective taking in understanding burnout in general practice" was published in 2014. Journal: BMC Fam Pract.

Experimental research has shown that the emotional load of being empathic could be regulated in trained individuals. For example, physicians have regulated negative affective arousal when confronted with the pain of others better than controls [24]. This regulation may have important benefits in freeing up cognitive resources necessary to help patients. This suggests that training in empathy could help physicians keep some distance in order to engage with their patients better, namely in a more cognitive fashion.

The interactional effect of perspective taking and empathic concern on burnout has potential important clinical implications. Our results suggest that there is no particular benefit in developing independent competencies for empathic concern, since when perspective taking abilities are not present, their protective impact on burnout is probably very limited. However, low perspective taking appeared to be negative irrespective of the level of empathic concern and as such, it merits being enhanced. When perspective taking abilities are present, it would be particularly recommended to develop empathic concern since both cognitive and affective empathy may interact to protect against burnout. Thus, it would be important to include both perspective taking and empathic concern into physicians’ training. Several studies have shown that these components of empathy could be influential and that their modification could impact physicians’ well-being, as well as their empathic behavior [21,40-42]. For example, training in mindfulness (i.e. training to focus more intently on the present moment with a sense of curiosity and openness) has been found to significantly improve perspective taking, physicians’ mood and well-being, while also decreasing burnout [41]. In a similar fashion, narrative training aims at developing the capacity to see things from others’ points of view and to reflect on one’s experience. This form of training has been shown to improve perspective taking and empathic concern on the IRI in physicians and other healthcare professionals [42].

It is important to note that the present study includes some limitations. First, we used a cross-sectional design, which did not allow for demonstration of causal relationships between empathy patterns and burnout. Indeed, several reports have underlined that burnout also erodes empathy [11,35,43]. One component of burnout, depersonalization, is partly defined as a lack of empathic attitudes. Future studies should develop strategies to control for this important aspect either statistically or by choosing more focused concepts, such as exhaustion or compassion fatigue. Second, our sample was not randomly selected. As a consequence, participants may not be representative of the population of general practitioners, which limits the external validity of the findings. Third, empathy and burnout were self-reported and consequently are subject to bias, such as social desirability. To overcome this problem, future research could use simple tasks to approach perspective taking [44].

The article "To be or not to be empathic: the combined role of empathic concern and perspective taking in understanding burnout in general practice" was published in 2014. Journal: BMC Fam Pract.

## Conclusions

Empathy is a crucial component of the patient-physician relationship. However, components of empathy are rarely examined in applied research. This is the first study to explore the interaction of cognitive and affective empathy to explain burnout in general practice. The present study’s findings suggesting a protective role of the interaction of cognitive empathy but not affective empathy alone may have implications in the design of curriculum interventions to promote general practitioners’ perspective taking and empathic concern and prevent burnout within this population. Teaching emotion regulation should also be included within the educational goals of health care professions, because without these skills physicians’ emotion sharing with patients could lead to professionals’ personal distress and burnout. Future research should focus on better understanding the interaction of perspective taking and empathic concern and its relationship to the mental health of physicians. Longitudinal studies will be necessary to determine the effect of empathy patterns on burnout over time, and subsequently to evaluate strategies of relating to others’ suffering more adequately.

## Competing interests

The authors declare that they have no competing interests.

## Authors’ contributions

ML participated in the design of the study, performed the statistical analysis and wrote the manuscript. EB co-designed the study and participated to data collection. FZ helped design the study, analyze the data and write the manuscript. SS designed and coordinated the study, found financial support and coordinated the writing of the manuscript. All authors read and approved the final manuscript.

## Authors’ information

ML is PhD candidate in health psychology, University of Montreal, Montreal, Canada.

EB is researcher in psychology, Paris Descartes University, France.

FZ is associate professor of psychology and researcher, Paris Descartes University, Paris, France.

SS is associate professor of pediatrics and psychology, University of Montreal, and senior researcher, Sainte-Justine UHC, Montreal, Canada.

## Pre-publication history

The pre-publication history for this paper can be accessed here:

http://www.biomedcentral.com/1471-2296/15/15/prepub
